The article "Effects of soot and plastic fibers on the performance of SCC" was retracted in 2024. Reason: duplicate publication.

# Effects of soot and plastic fibers on the performance of SCC

**DOI:** 10.1016/j.heliyon.2024.e36745

**Published:** 2024-08-29

**Authors:** Ali Sadrmomtazi, Nasim Sadat Ekrami

**Affiliations:** Department of Civil Engineering, Faculty of Engineering, University of Guilan, Rasht, Iran

**Keywords:** Self-compacting concrete, Iron oxide, Plastic belt fibers, Compressive strength, Tensile strength

## Abstract

Self-compacting concrete is regarded as one of the newest types of concrete due to its durability, efficiency, viscosity, stability, flowability, and resistance. Today, one of the most pressing environmental challenges is the disposal of solid waste, and one of the plastic materials discarded as waste after use is plastic packaging belts. These are made on the basis of polypropylene, as well as the factory Iron smelting mines are the main source of iron oxide waste production. Studies using recycled plastic fibers (30 mm × 0.3 mm) and waste iron oxide as cost-effective additives in self-compacting concrete (SCC) are presented. The effects on fresh and hardened properties were evaluated at various additive contents. Fresh and hardened properties of self-compacting concrete (SCC) were evaluated with and without fiber and iron oxide additives. Tests included workability (slump flow, funnel), strength (compressive, tensile), and durability (ultrasonic pulse speed, permeability). Experiments revealed that increasing the amount of recycled plastic fibers and waste iron oxide in self-compacting concrete (SCC) led to higher compressive and tensile strengths at both 7 and 28 days. These strength increases ranged from 2 to 9.68 MPa for compressive strength and 1.61–7.44 MPa for tensile strength, compared to the control specimen without additives.

## 1 Introduction

Self-compacting concrete can easily flow through all kinds of complex shapes or shapes that have many reinforcing bars, and due to its plasticity, does not cause porosity [1,2]. This type of concrete has low yield stress, high deformability, separation resistance and medium viscosity. Self-compacting concrete is more efficient in terms of flow and efficiency than ordinary concrete and they easily fill the entire form without vibration and has the ability to self-level on the surface [3]. It is usually better than regular concrete in terms of time, workability and durability. The ratio of water to cement in self-compacting concrete is lower than conventional concrete, and it obtains its fluid properties with superplasticizers and enhancing additives [4]. As a result, the use of self-compacting concrete is better and more efficient than conventional concrete. One of the important characteristics of self-compacting concrete is its viscosity and stability compared to other types of concrete [5]. Furthermore, because self-compacting concrete compresses under its own weight, it can be regarded as a cost-effective material to minimize installation costs, time, and vibration. Nowadays, mining and industrial activities produce much waste; this waste is generally buried because it is not or is little used [6].

One of the primary and significant issues with environmental pollution and natural resources, industry, and mining is the quantity of solid waste produced, which includes waste from industries, plastic material manufacturing companies, iron smelting companies, and mineral processing activities. As a result, strategies to reuse industrial waste have been developed. Over the past 20 years, there has been a surge in the use of industrial waste as building materials for embankments of roads, railroads, concrete, and dams rather than natural sand. Additionally, numerous researchers have looked into the possibility of using industrial solid waste to partially replace cement in concrete [7].

Natural sand and gravel are decreasing due to the increase in consumption in all types of concrete, and as a result, the replacement of natural sand and gravel as using waste has increased. One of the industrial wastes produced from steel and ingots in iron smelters is iron oxide (${Fe}_{2}O_{3}$), which appears during the cooling and hardening of steel ingots from the molten state, moisture and cooling in the dehumidifier. The main cause of this issue is the amount of moisture in the steel and its evaporation from the steel surface. It is also produced as a result of the steel surface's expansion and contraction, and it is regarded as trash once it has been cleaned off. Particles of iron oxide are smaller than those of cement. Due to its chemical makeup, iron oxide exhibits remarkable mechanical and physical qualities. Iron oxide forms a strong bond with Portland cement and adds great stability to the concrete mixture because of its soft texture and component composition [8]. Worldwide, massive amounts of iron oxide are wasted. Iran produces about 10,000 tons of iron oxide annually [9]. As iron oxide production continues to rise, it can be utilized in cement mixtures and concrete to improve resistance and durability rather than being disposed of in the environment. Additionally, it enhances the microstructure of concrete and helps to fill in the internal pores. It influences the mechanical characteristics of cement in self-compacting concrete because of its poor pozzolanic reactivity. Given that larger particle size aggregates (like sand and gravel) increase porosity, pores between particles, and inhomogeneity in the mixture, iron oxide is also used to improve homogeneity, compaction, reduce porosity, bulkiness, and resistance in order to achieve mechanical properties and durability of concrete. Using iron oxide extensively lowers the threats to the environment and natural resources [10].

The development of industry, technology, and population growth have all contributed to an increase in the production of solid waste, particularly plastics. Nowadays, plastics are used extensively in almost every facet of daily life [11]. But because plastics do not decompose, disposing of discarded ones has become difficult. Packaging waste makes up the majority of plastic waste. Wastes from plastic packaging are regarded as one of the environmental pollution sources. A significant threat to the environment and natural resources is posed by the fact that 70 % of packaging materials are disposed of in landfills, 20 % are burned, and just 7 % are recycled each year. Thus, using plastic packaging bags as leftover and recycled material in concrete also helps to recycle and conserve energy and production processes, as well as lessen environmental pollution. When used in place of some of the cement in the design of a concrete mix, plastic packing bags can be a useful way to address environmental issues [12]. It contributes to the enhancement of concrete's mechanical qualities because of its low density, chemical resistance, high modulus of elasticity, tensile properties, and thermal insulation when compared to other recycled materials. One of the best ways to dispose of plastic packaging belts is to incorporate them into concrete as fibers, which also increases the material's strength, ductility, and durability [13].

Various researches have been conducted in relation to the use of plastic packaging materials and iron oxide in concrete, some of which have been examined below. Singh and Siddique [2] in 2016 investigated the effect of iron slag as a partial replacement of fine aggregates on the durability characteristics of self-compacting concrete. The result of the experiment shows that self-compacting concrete containing iron slag has better durability than the control mixture of self-compacting concrete. Singh and Siddique [3] in 2016 investigated and analyzed the microstructural mechanical properties of self-compacting concrete with iron slag as a partial replacement of fine aggregates. The results showed that the compressive strength, tensile strength and bending strength of self-compacting concrete containing iron slag improved at all ages. SEM and XRD analysis were performed to investigate the microstructure, which showed that the use of iron slag makes the microstructure of self-compacting concrete denser.

Largeau et al. [4] in 2018 investigated the effect of iron powder (${Fe}_{2}O_{3}$) on the strength, performance and porosity of concrete. The results showed that the compressive and tensile strength changes up to 5 % with the replacement of iron powder. The efficiency of fresh concrete decreased with increasing amount of iron powder. Porosity was reduced by replacing 1.5 % and 2.5 % by weight.

Askari Dolatabad and Jahanshahi [6] in 2019 investigated the rheological and mechanical properties of lightweight self-compacting concrete containing Sirjan iron mine waste. The replacement of 5 % and 10 % by weight of cement with iron mine waste led to an increase of 8.6 % and 20 % in compressive strength compared to the control sample, respectively.

In 2019, Ismail Al-Hadithi et al. [7] investigated the mechanical and behavioral properties of self-compacting concrete reinforced with PET fibers. Experiments showed that the inclusion of PET fibers in self-compacting concrete leads to an increase in compressive and bending strength. A significant improvement in impact load resistance and energy absorption capacity of concrete with PET fibers was observed.

Zhao et al. [10] in 2021 investigated the use of iron waste in high-performance concrete and determined new properties and compressive behaviors of concrete. The results showed that the efficiency of concrete decreases with the increase of iron waste. The reduction in compressive behavior is mainly due to the loss of flowability.

Jaskowska et al. [11] in 2022 investigated the selected properties of self-compacting concrete with recycled PET. This research showed that both flow properties and properties of concrete hardened with PET are reduced. The compressive strength of concrete decreased by approximately 50 %. One of the most important components in the production of science is to consider the approach of sustainable development and improvement. Sustainable development is important with the concept of using the potential and available facilities in order to optimally use the available resources.

Faraj et al. [14] discussed the use of recycled plastic waste (RP) as a sustainable alternative in self-compacting concrete (SCC). Based on the results, recycled plastic self-compacting concrete (RPSCC) demonstrated satisfactory fresh properties (workability, flowability) as well as acceptable mechanical properties (strength) for structural applications. Besides, it was observed that replacing natural aggregates (NA) with RP contributed to a more environmentally friendly and sustainable concrete solution.

Hussain et al. [15] explored the use of recycled waste materials like glass and ceramic in the form of nanoparticles (NWM) as a partial replacement for cement in SCC. This approach aims to be more eco-friendly by reducing reliance on traditional cement production and utilizing waste materials. Conclusively, it was understood that using recycled waste materials in the form of nanoparticles as a partial cement replacement in SCC has promising potential for sustainable construction. While some workability challenges exist, the benefits in strength, microstructure, and potentially corrosion resistance make it a viable option for further exploration.

Hamza et al. [16] analyzed the effects of adding recycled steel fibers recovered from waste tires (SFR) on the properties of SCC. They prepared five SCC mixtures with varying SFR content from 0 to 1.5 %. They concluded that incorporating recycled steel fibers from waste tires can improve the SCC's resistance to bending (flexural strength) and reduce shrinkage. However, it comes at the cost of decreased workability (fresh properties) and potentially slightly lower compressive strength. The optimal content of SFR needs to be balanced based on the desired properties for a specific application.

Del Angel et al. [17] investigated the possibility of replacing natural sand with used foundry sand in SCC. For this purpose, they produced SCC mixes with two replacement levels for natural sand:

•50 % replacement with used foundry sand
• 100 % replacement with used foundry sand

Eventually, they found that replacing natural sand with used foundry sand, especially at high replacement levels (up to 100 % in this case), can be a sustainable alternative for SCC production. It offers improved fresh properties and significantly increased compressive strength, although some trade-offs might exist in splitting tensile strength.

Busic et al. [18] examined the effects of using recycled waste tire rubber as a replacement for natural aggregate in SCC. They produced seven concrete mixtures:

•One reference mix with only natural aggregate.
•Six mixes with waste tire rubber replacing 5 %–30 % of the total aggregate volume (maximum rubber size 4 mm).

They discovered that incorporating waste tire rubber up to a specific content (10 % in this case) can be a viable option for sustainable SCC production without compromising its performance.

Khoshakhlagh et al. [19] investigated the effect of adding iron oxide nanoparticles (Fe_2_O_3_) to high-performance self-compacting concrete (SCC). They studied the concrete's compressive strength, flexural strength, split tensile strength, and water absorption. Overall, they suggested that incorporating Fe_2_O_3_ nanoparticles within a specific content range can enhance the performance of high-performance SCC.

The innovative aspect of this research is in the direction of optimal use of waste resources and minimizing waste and environmental pollution. In order to increase tensile and compressive strength in self-compacting concrete, plastic packing fibers and oxide were used. In the self-compacting concrete mixing plan, nano silica gel and VMA were used to increase the strength, strengthen the transition zone of concrete (third phase), strengthen the increased viscosity and increase the rheological properties of concrete. The difference between this research and the other projects is that the permeability test, the effect of temperature on compressive strength, ultrasonic pulse speed and Schmidt hammer were also evaluated for the cubic samples of self-compacting concrete with and without iron oxide waste and plastic packaging fibers. The rheological and mechanical properties of self-compacting concrete containing iron oxide waste and plastic packaging fiber waste as an alternative to sand and cement were presented and discussed in this paper. The purpose of adding (IOW) and (PPFW) in the design of self-compacting concrete mix is to improve and increase tensile and compressive strength.

## 2 Laboratory program

### 2.1 Consumable materials

#### 2.1.1 Cement

Given that self-compacting concrete has a lower volume of cement paste than conventional concrete, selecting the right cement is critical. In this study, type 2 Portland cement supplied by Behbahan Cement Factory used for all five mixture designs, in accordance with the ASTM C150 standard [20] (see Table 1, Table 2).

**Table 1:** Chemical characteristics of type 2 Portland cement.

Chemical analysis	Percentage
IR^1^	0.24
SiO_2_	21.68
Al _2_O_3_	4.82
Fe_2_O_3_	3.88
CaO	65.4
MgO	2.08
SO_3_	0.68
Na_2_O	0.25
K_2_O	0.88
LOI	0.2
C_3_S	60.63
C_2_S	16.46
C_3_A	6.21
C_4_AF	11.8
Free Cao	0.7

**Table 2:** Mechanical characteristics of type 2 Portland cement.

Specifications	Amount
Softness of cement (blain) $\left({cm}^{2}/g\right)\left(BF\right)$	3220
Initial setup time (min) (IST)	155
Final setup time (min) (FST)	270
3-day compressive strength $\left(kg/{cm}^{2}\right)$	240
7-day compressive strength $\left(kg/{cm}^{2}\right)$	300
28-day compressive strength $\left(kg/{cm}^{2}\right)$	446

#### 2.1.2 Plastic packing belt fibers

Plastic belt (polyethylene terephthalate) is a durable and ideal material for packing industrial items. Polyethylene terephthalate is one of the most often used types of plastic belts, which are manufactured on highly advanced production lines. Polyethylene terephthalate is produced from recycled plastic bottles. Polyethylene terephthalate, a thermoplastic polyester resin, has the chemical formula (C_10_H_8_O_4_)_n_. This resistant material is used in various industries such as bottling, making plastic sheets and packing belts. These belts have many uses and features, among them high tensile strength, density and low weight compared to metal packaging belts, high resistance to temperature, non-toxic, environmentally friendly, impact and pressure. In fact, polyethylene terephthalate belt is recyclable and can also be produced from recycled materials. When the plastic belt is stretched between 20 and 40 % of its tensile strength, it has an increase in length between 2 and 6 % in the standard state. To produce this product, five steps are performed, which are: extrusion, stretching, ribbing of the belt, fixing and winding. In the first stage, granules (primary materials) and additives are granulated and refined and placed in the tank of the extrusion machine. While passing through this device, these materials are melted and passed through the extrusion molds and then pass through the water tubs to cool and solidify. In the tensioning stage, they continue the belt tensioning process until reaching the desired tension level. After that, to increase the strength of the belt, treads are made on it. Increasing the stiffness of the belt improves the feeding process (belt feeding or shooting) in belt tensioning devices. In the fixing stage, the belts are stabilized in a duct with heat, in the desired size, and the products are cooled again so that they do not change shape again. The tread of the belt causes the performance of the belt to improve by increasing its strength and reducing the friction of the belt surface. In this design, plastic packaging belt fibers with a thickness of 0.2 mm were cut with a length of 30 mm and a width of 0.3 mm and were used in the weight amount of cement in self-compacting concrete (according to Table 3 and Fig. 1).

**Table 3:** Characteristics of plastic packaging belt fibers.

Specifications	Amount
Modulus of elasticity (GPa)	9.5
Special Weight ($gr/{cm}^{3}$)	0.71
Water absorption (24 h)	0.09 %
Tensile Strength (GPa)	8.2
Shrinkage	0.09 %
Elongation at failure	41 %
Elongation in yielding	3 %
Melting Temperature (C)	194
Length (cm)	3
Thermal bending Temperature (C)	80

**Fig. 1:** a) Plastic packing belt fibers b) Size of plastic packing belt fibers.

#### 2.1.3 Iron oxide

Iron and oxygen combine chemically to form iron oxide. There are roughly sixteen different varieties of hydroxide and iron oxide combined. Oxyhydroxides and iron oxides are abundant in nature and are crucial to numerous biological and geological processes. There are two ways to obtain iron oxide: synthetic and mineral. Combinations of one or more iron oxides or iron combined with impurities like manganese, clay, or organic matter are referred to as natural iron oxides. Several methods can be used to create synthetic iron oxide. The method of producing iron oxide is synthetically in Foulad and Zob Ahan Company. In the steel and ingot production factory, after the moisture is finished and the steel is cooled by the cooling device, due to the temperature change in the steel particles and the rate of evaporation of the surface water in the steel, iron oxide is formed on the surface of the ingot (according to Fig. 2). The widespread use of iron oxide in various industries can lead to negative environmental consequences. Air and water pollution due to suspended particles and waste materials from iron oxide production processes has become one of the main concerns in this field. For this reason, proper control and management of waste and its emissions is of particular importance. Iron oxide (${Fe}_{2}O_{3}$) constitutes nearly 45 % of ingot and steel production. This oxide is black, dark brown and grey in color. The characteristics of iron oxide as a disposable material are: High resistance to color change in sunlight and stable in environmental conditions. By combining cement, it can make the surface of concrete more uniform. The combination of cement with iron oxide can also increase the resistance of alkaline materials, and also give more shine to the surface and increase the resistance of the cement paste. The main components of iron oxide are; Silicon dioxide (${SiO}_{2}$), aluminum oxide (${Al}_{2}O_{3}$), calcium oxide (CaO), magnesium oxide (MgO) and iron oxide III (${Fe}_{2}O_{3}$) are 95 % of the composition. Using iron oxide in making concrete is a good solution to remove it, which has a direct effect on the setting of cement and causes it to set quickly and increase the strength of cement. For the use of iron oxide in self-compacting concrete, sieve passed with number 30 was used (according to Fig. 2, Fig. 3 and Table 4, Table 5).

**Fig. 2:** a) Iron oxide (soot) b) Granulation of iron oxide from different sieves.

**Fig. 3:** Vicat needle test of cement with and without iron oxide.

**Table 4:** Vicat test results of cement with and without iron oxide.

Specifications	Time Setting (min)	Needle size (cm)
Portland cement type 2	1	2.8
Portland cement type 2 + iron oxide	1	1.5

**Table 5:** Characteristics of iron oxide.

Specifications	Modulus of elasticity (GPa)	Special Weight ($gr/{cm}^{3}$)	Water absorption (24 h)	Tensile Strength (GPa)	Melting Temperature (C)
Amount	183	5.27	151 %	810	3210

#### 2.1.4 Aggregates

Coarse aggregate (gravel) with a maximum size of 12.5 mm and sand with a maximum size of 2.36 mm were used in this mixed design. The sand and gravel used in this mixing plan was obtained from Ramhormoz, Khuzestan. Sand and gravel (peas, almonds) were granulated using suitable sieves. For the pea gravel passed through the $\frac{3}{8}$ sieve, the almond gravel passed through the $\frac{1}{2}$ sieve, and the sand passed through the 8 sieve were used, which is based on the ASTM C33 standard [21] (according to Table 6).

**Table 6:** Characteristics of aggregates.

Specifications	Sand water absorption	Water absorption of Pea sand	Water absorption of almond sand
Amount (%)	2.2	0.8	0.9

#### 2.1.5 Super lubricant and nano-silica gel

In order to achieve the desired efficiency in mixtures, due to the effect of excess water on concrete, it leads to water loss, separation and resistance. It is very important to use and choose the type of lubricant to reduce the negative effect of too much water on the properties of fresh self-compacting concrete. Several main factors are important in choosing the type of lubricant, including efficiency, dosage and compatibility with Portland cement. In this research, in order to achieve the mechanical properties of self-compacting concrete, SUPER PLAST PC5000, which is based on polycarboxylate, was used as a type of reducing water and a very strong concrete enhancer. Also, in order to achieve rheological properties in the pasty state and to improve the quality of self-compacting concrete, nano-silica was used, which is based on silica fume and is a strong reducer of concrete water. Using nano silica improves the concrete's compressive strength, lowers its permeability, and makes concreting easier by making the concrete more efficient and slumping more. Additionally, according to ASTM C 494 standard [22], nano silica can influence the ultimate strength of concrete and strengthen the transition zone (third phase) (according to Table 7).

**Table 7:** Technical specifications of super-lubricant and nano-silica.

Physical Condition	Specific gravity (kg/l)	PH	Color
Super Lubricant SUPER PLAST PC5000			
Liquid	1.1	6.2	Yellow
Nano Silica			
Thick Liquid	1.35	9	Grey

#### 2.1.6 Water

In compliance with ASTM C 94 standard [23], drinkable water was used in the design of the self-compacting concrete mix for sample manufacture and processing (see Table 8).

**Table 8:** Characteristics of drinking water.

Specifications	Temperature (C)	PH	Chloride ion concentration
Amount	20	6	50

#### 2.1.7 Limestone powder

Stone powder is one of the ingredients required to guarantee the right viscosity in self-compacting concrete. Because they contain very small particles, fillers like stone powder cover the spaces between the aggregate and cement particles, decreasing porosity and increasing the degree of bulkiness in the concrete. Because this type of filler element has a very high specific surface area, it enhances the friction between the grains and the viscosity of the concrete. The results of chemical analysis of limestone powder are shown in Table 9. In this design, Qom limestone powder was used. As can be seen from Table 9, the main constituents of limestone powder used are SiO_2_, Al_2_O_3_, Fe_2_O_3_, MgO, Cao and SO_3_, which Cao is the most common constituent of limestone powder, which is equal to 51.22 %.

**Table 9:** Qom limestone powder.

Chemical Analysis	SiO_2_	Al_2_O_3_	Fe_2_O_3_	MgO	Cao	SO_3_	L.O.I
Percentage	2.8	0.35	0.5	1.8	51.22	1.24	43.2

#### 2.1.8 Concrete rheology thickener and controller

Increased viscosity and regulated rheological characteristics are produced in self-compacting concrete with the use of VMA powder additive. The management of surplus water in concrete is mostly dependent on VMA. The Master Matrix VMA 358 additive, which is based on heavy polymer molecular strands with exceptional stability, was employed in this study. As per the ASTM C 494/C 494M standard [24], the quantity of this ingredient in the concrete mix design is determined based on the weight of cement (Fig. 4).

**Fig. 4:** Materials used in self-compacting concrete mixing plan. 1-sand, 2-pea sand, 3-almond sand, 4-stone powder, 5-water, 6-superlubricant,7-nano silica gel, 8-viscosity modifier additive, 9-cement.

### 2.2 Mixed design

This study looked at five different self-compacting concrete mixing systems both with and without the addition of iron oxide and plastic packing belt fibers. In relation to the weight of cement, the percentage of plastic packing belt fibers is 0, 0.5, 1, 1.5, and 2 %; in relation to the weight of gravel, it is 0, 5, 10, 15, and 20 %. Because test findings are more transparent and reliable, all five mixed designs have the same amount of materials but different percentages of plastic packing belt fibers and iron oxide (Table 10).

**Table 10:** Mixing design of self-compacting concrete with and without plastic packing belt fibers and iron oxide.

Cement $kg/m^{3}$	Pea sand $kg/m^{3}$	Almond sand $kg/m^{3}$	Sand $kg/m^{3}$	Water $kg/m^{3}$	Super lubricant – micro silica super gel $kg/m^{3}$	Stone powder $kg/m^{3}$	VMA $kg/m^{3}$	Plastic packing belt fibers $kg/m^{3}$	iron oxide $kg/m^{3}$
Mixing design of self-compacting concrete without plastic packing belt fibers (0 %) and iron oxide (0 %) (SCC)									
500	350	140	1067	154	7–12	207	0.167	–	–
Mixing design of self-compacting concrete with plastic packing belt fibers (0.5 %) and iron oxide (5 %) (SCC FO1)									
500	350	140	1067	154	7–12	207	0.167	2.5	24.5
Mixing design of self-compacting concrete with plastic packing belt fibers (1 %) and iron oxide (10 %) (SCC FO2)									
500	350	140	1067	154	7–12	207	0.167	5	49
Mixing design of self-compacting concrete with plastic packing belt fibers (1.5 %) and iron oxide (15 %) (SCC FO3)									
500	350	140	1067	154	7–12	207	0.167	7.5	73.5
Mixing design of self-compacting concrete with plastic packing belt fibers (2 %) and iron oxide (20 %) (SCC FO4)									
500	350	140	1067	154	7–12	207	0.167	10	98

### 2.3 Performing the test

To conduct the test, the aforementioned components were combined for 10 min. The slump flow test, V funnel test, L box test, J ring test, and U box test must be performed for the qualities of fresh concrete (self-compacting with and without plastic packing belt fibers and iron oxide) after the components have been mixed in the mixer.

#### 2.3.1 Slump flow test

Slump flow test is very common to determine the performance of self-compacting concrete due to its simplicity. The results of the slump flow test of self-compacting concrete with the effect of different percentages of plastic packaging belt fibers and iron oxide in Fig. 5 are obtained based on the average.

**Fig. 5:** a) Slump flow test b) Slump flow test results.

The results of the slump flow test showed that with the increase in the percentage of plastic packing belt fibers and iron oxide, the slump diameter (flowability) decreased by 6.57, 9.21, 13.15, and 17.17 % respectively compared to self-compacting concrete (standard). It was found that the slump flow time was increased by 0.8, 1.4, 1.9, and 2.8 s respectively compared to self-compacting concrete (standard), which test is in accordance with ASTM C1611 standard [25].

#### 2.3.2 Funnel test V

The V-funnel test is used to gauge how well self-compacting concrete can shift its flow direction and go through bound and reinforced areas without causing the grains to separate and obstruct the flow. Based on averages, the V-shaped test results of self-compacting concrete in Fig. 6 with the impact of varying percentages of iron oxide and plastic packaging belt fibers were produced.

**Fig. 6:** a) V-funnel test b) V-funnel momentary test c) V-funnel 5-min test.

The results of momentary test and 5 min test of V funnel showed that with the increase in the percentage of plastic packaging belt fibers and iron oxide, the time was 0.9, 1.6, 2.5, 3.1 and 1.1, 1.8, 2.5, 3.9 s increased compared to the self-compacting concrete (standard) respectively, the tests are in accordance with the ISISIR 3203-9 standard [26].

#### 2.3.3 L box test

The L box test is used to evaluate the concrete's flowability, filling ability, stability against grain separation, and power transfer between rebars. Based on the average, the test results of the L box of self-compacting concrete in Fig. 7 with the impact of various percentages of iron oxide and plastic packing belt fibers were obtained.

**Fig. 7:** a) L box test b) L box test results.

The results of the L box test showed that with the increase in the percentage of plastic packaging belt fibers and iron oxide, the time was increased by 0.3, 1, 1.5, and 2 s, respectively, compared to self-compacting concrete, and the height of the concrete at the end of the horizontal section ($H_{2}$) and The end of the vertical section ($H_{1}$) was determined from the $H_{2}/H_{1}$, that with the increase in the percentage of plastic packaging belt fibers and iron oxide, the ratio of is 2.27, 5.68, 9.09, 11.36 decreased compared to self-compacting concrete, which is tested according to INSO 3203-10 standard [27].

#### 2.3.4 J ring test

The J-ring test is actually a simulation of the passage of concrete through rebars and is used to check the ability to pass. The test results of J-ring of self-compacting concrete with the effect of different percentages of plastic packaging belt fibers and iron oxide in Fig. 8 are obtained based on the average.

**Fig. 8:** a) J ring test b) J ring test results.

The results of the J-ring test showed that with the increase in the percentage of plastic packing belt fibers and iron oxide, the diameter of the slump (flowability) decreased by 4.41, 10.29, 14.70, and 19.11 %, respectively, compared to self-compacting concrete (standard). And the slump flow time also increased by 1.1, 2.2, 3, 4 s compared to self-compacting concrete (standard), which test is in accordance with INSO 11271 standard [28].

#### 2.3.5 U box test

It is employed to gauge how well self-compacting concrete fills and passes. This experiment uses a U-shaped container as its format. This device is made up of a moveable valve in the middle of a duct that is split into two sections by a dividing blade. The purpose of this test is to determine how well self-compacting concrete can fit through small web outlets below a specific height. Based on the base material, Fig. 9 shows the test results of the self-compacting concrete U-box with the influence of various percentages of packing belt fibers and iron oxide.

**Fig. 9:** a) U box test b) U box test results.

The results of the U box test showed that with the increase in the percentage of plastic packaging belt fibers and iron oxide, the time also increased, respectively, 0.6, 1.1, 2, 2.5 s compared to self-compacting concrete (standard) and the amount of concrete height difference in two ducts ($H_{2}-H_{1}$) it was increased by 1, 2, 3, 4 mm respectively compared to self-compacting concrete (standard). The difference in the height of concrete in the two ducts ($H_{2}-H_{1}$) was less than 30 mm and was accepted. The test is in accordance with UNI 11044 standard [29].

### 2.4 Molding of concrete samples

Fresh concrete was molded in cubic molds with dimensions of 150×150×150 mm and cylindrical molds with dimensions of 150×300 mm. The samples were kept at a temperature of 23 °C for 24 h to harden, and after 24 h, the samples were taken out of the molds and kept in the water basin for processing for 7 and 28 days. A total of 1000 samples of self-compacting concrete with and without plastic packing belt fibers and iron oxide were made, of which 500 samples were made in cubic form and 500 samples were made in cylindrical form. After 5 mixed designs reached the age of 28 days, Schmidt hammer test according to ASTM C805 standard [30], ultrasonic pulse speed test according to ASTM C-597 standard [31], permeability test according to DIN 1048 standard [32], temperature effect Regarding the compressive strength, compressive strength of the cubic specimens during 7 and 28 days of curing according to the ISIRI 3206 standard [33] and the tensile strength of the cylindrical specimens was performed according to the ASTM C496 standard [34]. A concrete breaker jack was used to break the specimens. Finally, after the Schmidt hammer test, the ultrasonic pulse velocity test and the failure of the specimens, the results of the specimens with self-compacting concrete (control) were compared and a correlation was established with the Schmidt hammer test and the ultrasonic pulse velocity.

### 2.5 Schmidt hammer test

Tests for the compressive strength of cylindrical and cubic specimens were performed using the Schmidt Hammer test. Concrete's compressive strength, in particular, can be determined with Schmidt's hammer when evaluating elastic material properties. Schmidt's hammer is now regarded as a non-destructive test and, because of its hardness, it has been utilized recently as an efficient instrument for surface resistance of objects [35]. In this way, the reliable reading and recording of the index number with the Schmidt hammer was done on the samples and the results were mentioned, which is in accordance with the ISO1920-7 standard [36] (according to Fig. 10, Fig. 11, Fig. 12). The results of the tests on cubic and cylindrical samples showed that by adding plastic packing belt fibers and iron oxide to self-compacting concrete, the compressive strength increased with the Schmidt hammer test. The reason for the increase in the Schmidt hammer test to measure the compressive strength for cubic and cylindrical specimens is due to the positive effect of the empty space filled with iron oxide in the self-compacting concrete due to the amount, shape and dispersion in the concrete. Also, the increase in the compressive strength of the samples with the increase in the percentage of fibers and iron oxide is due to the reduction of porosity due to the addition of iron oxide and, as a result, the increase in adhesion between cement and aggregates, the increase in adhesion in the concrete transition area and the sufficient cohesion of concrete.

**Fig. 10:** Schmidt hammer test on the specimen.

**Fig. 11:** The results of the Schmidt hammer test for the cube samples in 28 days processing.

**Fig. 12:** Schmidt hammer test results for cylindrical specimens in 28 days processing.

### 2.6 Ultrasonic pulse speed test

Ultrasonic pulse velocity testing is one of the non-destructive testing methods that determines the possibility of in-depth analysis of material homogeneity, uniformity, quality, wear, finding defects, the presence of internal cavities and voids in hardened concrete. The speed of ultrasonic waves in this research is in the frequency range of 20–170 kHz. Also, the direct method was used to conduct the test, and the distance between the two ultrasonic transducers is 150 mm for cubic samples and 300 mm for cylindrical samples, which is in accordance with the ISO1920-7 standard [36]. According to equation (1), the distance (cm) is divided by the reading number (ms) displayed on the device screen and multiplied by 10 to determine the pulse speed in (km/s). The criterion for determining the quality of concrete based on this test is obtained by controlling the wave speed in the specified standard intervals (km/s), and if its value is less than 3, the result is not favorable, and if it is higher than 3, the result is favorable and it is acceptable [37] In this way, the number of ultrasonic readings and the distance between the two transducers were performed on the samples and the results were noted (according to Fig. 13, Fig. 14, Fig. 15). The results of the tests on cubic and cylindrical samples showed that the speed of the ultrasonic pulse increased with the addition of plastic packing belt fibers and iron oxide to the self-compacting concrete. As can be seen, the ultrasonic pulse speed in SCC F01 to SCC F04 samples increased by 7.5, 25, 37.5 and 57.5 % in cubic samples and 12.5, 25, 37.5 and 50 % in cylindrical samples, respectively.

**Fig. 13:** Testing the speed of the ultrasonic pulse on the test piece.

**Fig. 14:** Ultrasonic pulse speed test results for cube samples in 28 days processing.

**Fig. 15:** Ultrasonic pulse speed test results for cylindrical samples in 28 days processing.

The reason for the increase in the test results of ultrasonic pulse speed on self-compacting concrete is due to the filling of empty space and the decrease of permeability in self-compacting concrete due to the amount, shape and dispersion of fibers and iron oxide in concrete. The results of the pulse speed test are also positively impacted by increasing the percentage of fibers and iron oxide in the samples because of the fibers' efficient absorption of water. Additionally, increasing the percentage of iron oxide decreases porosity, which increases adhesion between cement and aggregates, increasing the pulse speed in concrete by providing sufficient cohesion and adhesion in the concrete transition area.

(1) $$km/s=\frac{cm}{ms}\times 10$$

### 2.7 Penetration testing of cubic specimens

The permeability test of self-compacting concrete was considered for cubic specimens with dimensions of 150×150×150 mm to protect the specimens against water and the durability of concrete, which is of particular importance. Functionally, permeability is also closely related to the These days of concrete, especially its resistance to gradual deterioration under exposure to severe weather and settlement caused by water penetration, especially when it contains aggressive gases or minerals in solution. Permeability of concrete against water, corrosion caused by carbonation, etc. are among the most influential factors in the durability of concrete. Durability of concrete means its ability to deal with atmospheric factors, chemical attacks, wear, erosion and any process that leads to deterioration and deterioration and reducing its useful life and efficiency. Therefore, determining the permeability characteristics of self-compacting concrete is of considerable importance. This test was carried out for cubic specimens exposed to 5 bar hydrostatic pressure, which was measured according to DIN 1048 standard [26]. Water penetrates through concrete pores during a certain period of time and the permeability coefficient is calculated. The concrete permeability test was performed in a period of 72 h at a temperature of 27 °C.

Concrete's permeability can be effectively decreased by adding fibers and iron oxide. Due to their good mechanical qualities, fibers and iron oxide can aid in bonding and strengthening concrete components. As a reinforcing additive, iron oxide and fibers can assist reduce bursting and cracking and strengthen concrete. These two can decrease permeability and sealed materials in concrete while also improving the mechanical and physical qualities of the material. Concrete's internal structure, which includes its strength, flexibility, and water-permeation barrier, can be enhanced by the addition of fibers and iron oxide. In general, oxide and fibers can be used to improve the durability and decrease permeability of concrete. As can be seen from Fig. 16, by adding the amount of fibers and iron oxide, the permeability of concrete decreased. So that the reduction of permeability in the plan was SCC F04 to 38.8 % compared to the control sample.

**Fig. 16:** Concrete permeability device and permeability test results.

### 2.8 Testing the effect of temperature on the strength of cubic specimens

This experiment demonstrates the impact of varying temperatures on the atmosphere and the interior of self-compacting concrete with and without plastic packing belt fibers and iron oxide. In a cube mold, fresh self-compacting concrete samples with and without fibers and oxide are first formed. The molds are then placed in a furnace drier at varying temperatures, as shown in Fig. 17, Fig. 18. The molds were taken out of the oven after the samples had hardened for 24 h, and a 1-day compressive strength test was conducted with documented results. Because the self-compacting concrete has been placed in the oven for 24 h and operations in concrete such as temperature changes, heat of hydration in cement, thermal properties of self-compacting concrete, heat transfer from mold to self-compacting concrete, etc [3]. which significantly affect the stability and durability of concrete; Therefore, the 1-day compressive strength of self-compacting concrete was performed [38].

**Fig. 17:** a) Cubic specimen in the oven b) Specimen after leaving the oven c) Failure of the specimen with the compressive strength device.

**Fig. 18:** a) Testing the effect of temperature on 1-day compressive strength b) Testing the effect of temperature on permeability coefficient.

According to the experiment results, the 1-day compressive strength and permeability of five different designs of concrete mixes decreased as temperature increased. However, at 25 °C, when the percentages of plastic strapping fibers and iron oxide in self-compacting concrete increased, the 1-day compressive strength of the cubic specimens increased to the highest point, and the permeability of the specimens was lower than that of concrete without fibers and oxides.

### 2.9 Testing the compressive strength of cubic specimens

The compressive strength of 5 mixed designs based on the ages of 7 and 28 days with cubic dimensions of 150×150×150 mm were investigated. The test results on cubic specimens based on the ISIRI 3206 standard [33] showed that with the addition of plastic packaging belt fibers and iron oxide to self-compacting concrete, the compressive strength increases (according to Fig. 19, Fig. 20). The reason for the increase in the test of the compressive strength of the cubic samples is due to the positive effect of filling the empty space created by iron oxide, creating more adhesion of the aggregate with cement, the effect of the fibers due to the amount, shape and dispersion in the concrete. Also, increasing the percentage of iron oxide reduces the porosity and consequently increases the adhesion between cement and aggregates, increases adhesion in the transfer zone (third phase) of concrete and sufficient cohesion of concrete, the main reason for increasing concrete strength is the reaction between cement and it is iron oxide that helps the adhesion between coarse cement particles and coarse aggregate and makes the structure and mechanical properties of concrete durable.

**Fig. 19:** a) Compressive strength fracture test of cubic test piece with concrete breaker jack device b) Broken test piece of self-compacting concrete with fibers and iron oxide.

**Fig. 20:** a) Compressive strength test results for cubic specimens in 7-day processing b) Compressive strength test results for cubic specimens in 28-day processing.

As can be seen in Fig. 20, the average compressive strength of all samples is higher than the control sample, which increased with the increase in the amount of fibers and iron oxide. The greatest increase in the compressive strength of the samples at the age of 7 and 28 days is about 9.2 and 9.5 %, respectively.

### 2.10 Testing the tensile strength of cylindrical samples

The tensile strength of 5 mixed designs based on the ages of 7 and 28 days with cylindrical dimensions of 150×300 mm were investigated. The results of tests on cylindrical specimens based on the ASTM C496 standard [34] showed that the tensile strength increases with the addition of fibers and iron oxide to self-compacting concrete (according to Fig. 21, Fig. 22). The reason for increasing the tensile strength test in self-compacting concrete with iron oxide and fibers for cylindrical tests is due to the positive effect of the unique characteristic of plastic strapping fibers with respect to its tensile strength and modulus of elasticity in self-compacting concrete due to the quantity and size. and reduces cracking in concrete, also iron oxide increases adhesion between aggregate and cement in concrete. As can be seen, the tensile strength of SCC 401 to SCC F04 samples has increased by 12, 21, 41 and 58 % in cubic samples and 24.4, 39.3, 64.2 and 76.6 % in cylindrical samples, respectively.

**Fig. 21:** a) Tensile fracture test of cylindrical specimen with concrete breaker jack b) Broken specimen of self-compacting concrete with fibers and iron oxide.

**Fig. 22:** a) Tensile strength test results for cube samples after 7 days processing b) Tensile strength test results for cube samples after 28 days processing.

## 3 Data availability statement

No data was used for the research described in the article.

## 4 Conclusion

This study examined the application of iron oxide and plastic packing belt fibers to self-compacting concrete. This research has the potential to significantly lower the cost of materials and structures, lessen environmental pollution and its negative effects, increase the strength and tensile and compressive properties of concrete, preserve natural resources, and reduce brittleness and cracks in the material. The primary accomplishment of this article allows for the attainment of the following outcomes:

1) After 7 and 28 days of processing, the average compressive strength test results of self-compacting concrete cube samples with plastic packing belt fibers and iron oxide revealed that the addition of fibers and iron oxide resulted in 2, 3.79, 6.87, 9.68 % and 1.61, 3.28, 4.34, and 7.44 % increased strength, respectively, in comparison to the self-compacting concrete sample (control).
2) Following 7 and 28 days of processing, the average tensile strength test results of cylindrical samples of self-compacting concrete with plastic packing belt fibers and iron oxide revealed that the addition of fibers and iron oxide resulted in increased strength relative to the self-compacting concrete sample (control) of 14.37, 26.81, 44.61, 58.35, 21.09, 35.57, 57.95, and 72.57 %.
3) Using a return hammer and self-compacting concrete with plastic packing belt fibers and iron oxide over the course of 28 days of processing, the average results of the compressive strength test of cubic samples revealed that an increase in fibers and iron oxide was associated with increases in strength of 27.3, 5.09, 7.27, and 9.27 % when compared to the self-compacting concrete sample (control).
4) After 28 days of processing, the average compressive strength test results of cylindrical specimens using a return hammer on self-compacting concrete with plastic packing belt fibers and iron oxide revealed that the addition of fibers and iron oxide resulted in increases in strength of 1.38, 7.34, 9.92, and 13.69 % when compared to the self-compacting concrete sample (control).
5) The average results of the ultrasonic pulse velocity test on cubic samples of self-compacting concrete with plastic packing belt fibers and iron oxide over the course of 28 days of processing revealed that increases in pulse speed were observed in relation to the self-compacting concrete sample (control) with increases in fiber and iron oxide of 10, 25, 32.5, and 57.5 %.
6) During the course of 28 days of processing, the average results of the ultrasonic pulse speed test on cylindrical samples of self-compacting concrete with plastic packing belt fibers and iron oxide revealed that the presence of fibers and iron oxide increased the pulse speed of the sample by 14.28, 19.04, 23.8, and 33.33 % when compared to the self-compacting concrete sample (control).
7) When self-compacting concrete with plastic packing belt fibers and iron oxide was tested for its 1-day compressive strength over a period of time, the average results showed that the strength increased with the amount of fibers and iron oxide. The values found were 5.22, 9.15, 15.22, and 20.64 % when compared to the self-compacting concrete sample (control).
8) The effect of temperature on the 1-day compressive strength of self-compacting concrete with plastic packing belt fibers and iron oxide was tested on average results for cubic samples. The results showed that the strength increased with the amount of fibers and iron oxide; values were 5.22, 9.15, 15.22, and 20.64 % when compared to the self-compacting concrete sample (control).
9) The average results of the permeability test conducted on self-compacting concrete with plastic packing belt fibers and iron oxide for cubic samples over the course of a 28-day processing period revealed that permeability decreased in comparison to the self-compacting concrete sample (control) as fiber and iron oxide levels increased by 7.32, 15.96, 24.72, and 37.33 %, respectively.
10) The average results of evaluating the impact of spal on the one-day permeability of self-compacting concrete with plastic packing belt fibers and iron oxide for cubic samples revealed that permeability decreased in comparison to the self-compacting concrete sample (control) as fiber and iron oxide levels increased, with values of 8.33, 15.25, 21.83, and 29.82 %, respectively.
11) The maximum decreases in the permeability of samples is related to sample SCC F04, which decreased by 38.8 % compared to the control sample.
12) The average of the highest percentage increase in compressive strength compared to the control sample is related to sample SCC F04, which is 9.2 and 9.8 % at the age of 7 and 28 days, respectively

## CRediT authorship contribution statement

**Ali Sadrmomtazi:** Methodology. **Nasim Sadat Ekrami:** Investigation.

## Declaration of Competing interest

The authors declare that they have no known competing financial interests or personal relationships that could have appeared to influence the work reported in this paper.
